The article "Influences of Oral Administration of Probiotics on Posthepatectomy Recovery in Patients in Child-Pugh Grade" was published in 2022. Journal: Comput Math Methods Med.

# Influences of Oral Administration of Probiotics on Posthepatectomy Recovery in Patients in Child-Pugh Grade

**DOI:** 10.1155/2022/2942982

**Published:** 2022-07-08

**Authors:** Hao Huang, Fang Fang, Zheng Jia, Wen Peng, Yi Wu

**Affiliations:** Department of Nursing, Shanghai General Hospital, Shanghai 200080, China

## Abstract

**Objective:**

This study is aimed at investigating the influences of oral administration of probiotics on posthepatectomy recovery in patients in Child-Pugh grade.

**Methods:**

100 patients (50 cases in Child-Pugh A grade and 50 cases in Child-Pugh B grade) underwent hepatectomy in our hospital from January 2018 to January 2020 were involved in this study. Subsequently, Child-Pugh A grade and Child-Pugh B grade patients were set as probiotics group (taking Clostridium butyricum, *n* = 25) and control group (no probiotics, *n* = 25). The general information, infectious indexes, and liver function indexes on days 1, 3, and 5 after operation were collected.

**Results:**

In Child-Pugh B grade subgroup patients, the procalcitonin, alanine aminotransferase, and prothrombin time of the probiotics group were statistically significantly lower than that of the control group on days 3 (*P* < 0.05) and 5 (*P* < 0.05) after surgery. In Child-Pugh A grade subgroup patients, there were no significant differences between probiotics group and control group after operation.

**Conclusion:**

Child-Pugh A grade subgroup patients with hepatectomy could not benefit from oral probiotics. However, Child-Pugh B grade subgroup patients taking probiotics after hepatectomy could reduce postoperative infection and accelerate recovery of liver function.

## 1. Introduction

Partial hepatectomy is a pivotal method of treating benign and malignant liver tumors that can effectively reduce the mortality of patients and improve their quality of life [1]. But patients are prone to suffering from the abdominal, incisional wound, and urinary system infections after surgery, due to liver dysfunction and body immunity reduction, which increases the pain and affects patients' recovery. Meanwhile, patients are at risk for adverse outcomes such as prolonged hospitalization stays, extra medical costs, and increased mortality [2–4].

Recent attention has focused on the relationship between gut-microbiota-liver axis and the intestinal flora and its pathological significance. Small amount of endotoxin produced by the intestinal flora enters the liver through the portal system and is phagocytosed and cleared by hepatocytes under physiological conditions. And liver dysfunction can cause reduced body immunity, alteration of intestinal flora, and increased endotoxin level, leading to aggravation of hepatocyte damage and formation of a vicious circle [5, 6]. Clinical research and animal experiments both presented potential clinical application of probiotics in hepatic injury caused by alcoholic hepatitis or fatty liver [7–9]. Probiotic preparations are ecological preparations made from normal microorganisms that are beneficial to the host or their microbial growth-promoting substances, which can effectively adjust intestinal flora alteration, restore the intestinal microecological environment, repress the excessive reproduction of Gram-negative (G-) bacilli, and decrease serum endotoxin level [10, 11]. Furthermore, probiotics have been used prophylactically to prevent bacterial infections after abdominal surgery [12]. Clinical trials also manifest that the bacterial infections after pancreatic surgery, hepatectomy, and liver transplantation can be reduced by prebiotics and probiotics (synbiotics) [13–15].

The article "Influences of Oral Administration of Probiotics on Posthepatectomy Recovery in Patients in Child-Pugh Grade" was published in 2022. Journal: Comput Math Methods Med.

Preoperative Child grading is a quantitative grading standard for evaluating liver reserve function in patients with liver disease and can indicate the severity of liver damage [16]. Patients in Child-Pugh C grade who underwent partial hepatectomy are implicated in high death rate and complication rate [17]. Thus, patients with Child-Pugh C grade were not included in this study, although Child-Pugh C grade is now no longer a contraindication to surgical treatment [18]. In this study, we investigated the impact of preoperative oral Clostridium butyricum on postoperative infection and recovery of liver function in patients in Child-Pugh A grade and Child-Pugh B grade after partial hepatectomy.

## 2. Objects and Methods

### 2.1. Research Objects

100 patients underwent partial hepatectomy in Shanghai General Hospital from January 2018 to January 2020 were collected, including 80 males and 20 females with a mean age of 50.3 years (25-75 years). 92 patients were diagnosed with primary liver cancer, and 8 patients were diagnosed with hepatic hemangioma preoperatively. According to the preoperative Child classification (see Table 1), 50 cases were in grade A and 50 cases were in grade B.

Patients who met the following inclusion criteria were deemed eligible for inclusion: (1) patient underwent partial hepatectomy; (2) patient did not have infection before surgery; (3) patient is older than 18 years old; (4) patient did not take probiotics in the past 1 week; (5) patient signed the informed consent. Patients who were not conforming to the inclusion criteria were excluded, detailed as follows: (1) patient had chronic constipation or diarrhea; (2) patient had liver function failure due to excessive liver resection, without postoperative complications such as bile leakage and massive bleeding; (3) patient underwent hepatic enterostomy or choledochojejunostomy; (4) patient had poor compliance; (5) patient had mental disorders.

The article "Influences of Oral Administration of Probiotics on Posthepatectomy Recovery in Patients in Child-Pugh Grade" was published in 2022. Journal: Comput Math Methods Med.

### 2.2. Grouping and Treatment

Patients in grade A/B were randomly grouped into probiotics group (*n* = 25) and control group (*n* = 25). Patients in the probiotics group received Clostridium butyricum (MIYAIRI, Japan) 3 × 2 tablets daily for three consecutive days before surgery. Prior to surgery, the patients were put on a 12 h fasting and 6 h water fasting. Then, the Clostridium butyricum was taken for 4 days after surgery. In the contrast, patients in the control group did not receive probiotics. This research protocol received approval from the Ethics Committee of Shanghai General Hospital, and all patients signed the written informed consent.

### 2.3. Data Collection

Baseline parameters of patients were as follows: sex, age, body mass index (BMI), presence or absence of liver cirrhosis, serum total bilirubin (TBIL), serum albumin (ALB), coagulation index (prothrombin time (PT)), and surgical method.

Detection indexes on days 1, 3, and 5 after surgery were as follows: fasting blood samples from each patient and healthy subjects were collected. Their infection indexes (procalcitonin, limulus test for endotoxins, and interleukin-6 (IL-6)) and liver function (alanine aminotransferase (ALT) and TBIL) were detected. Procalcitonin and IL-6 were measured by procalcitonin and IL-6 ELISA kit, respectively. Endotoxin levels in patients were detected using a chromogenic LAL assay kit (Lonza, USA) according to the manufacturer's instructions. Liver function indexes and coagulation indexes were assessed using Roche Cobas 8000 automatic biochemical analyzer (Roche, Germany).

### 2.4. Statistical Methods

Statistical analysis was processed by GraphPad Prism 5.0 (GraphPad Software Inc., San Diego, CA, USA). Measurement data were presented as mean ± SD, and a statistical comparison between the two groups was done by means of the *t*-test. Enumeration data were shown as numbers and percentages and were analyzed by Fisher's exact test or Pearson's *χ*^2^ test. Statistical significance was set at *α* = 0.05.

## 3. Results

### 3.1. Comparison of Baseline Information of Patients

There were 50 cases both in Child-Pugh A grade and Child-Pugh B grade. In the two subgroups, no statistically significant differences in sex, age, and BMI were observed between the probiotics group and the control group (Table 2). With regard to liver conditions, we found no statistically significant differences in presence or absence of liver cirrhosis, serum TBIL, and serum albumin index between the results. Moreover, there was also an absence of statistically significant differences in PT (a coagulation index indicating liver synthesis function), creatinine (a renal function index), and surgical method.

The article "Influences of Oral Administration of Probiotics on Posthepatectomy Recovery in Patients in Child-Pugh Grade" was published in 2022. Journal: Comput Math Methods Med.

### 3.2. Comparison of Infection Indexes of Patients

The following infection indexes were selected: procalcitonin is a specific index of severe bacterial inflammation and fungal infection and is associated with sepsis; limulus test for endotoxins indicates is used to reflect G-bacterial infection; IL-6 is an index that reflects early infection. The specific information of infection indexes is listed in Table 3.

In Child-Pugh A grade subgroup, there were no statistically significant differences in procalcitonin, limulus test for endotoxins, and IL-6 between the probiotics group and the control group on days 1, 3, and 5 after surgery.

In Child-Pugh B grade subgroup, the procalcitonin in the probiotics group and the control group on day 3 after surgery was 0.80 ± 0.96 and 1.98 ± 1.88, respectively, with a statistically significant difference (*P* = 0.007). The procalcitonin levels in the probiotics group and the control group on day 5 after surgery were 0.29 ± 0.47 and 1.14 ± 1.59, respectively, with a statistically significant difference (*P* = 0.014). These observations suggested that the postoperatively early bacterial infection rate in the probiotics group was lower than that in the control group.

### 3.3. Comparison of Liver Function Recovery Indexes in Patients

In the Child-Pugh A grade subgroup, there were no statistically significant differences in ALT, TBIL, and PT between the probiotics group and the control group on days 1, 3, and 5 after surgery.

In the Child-Pugh A grade subgroup, the ALT and the PT of the probiotics group were statistically significantly lower than that of the control group on days 3 and 5 after surgery (*P* < 0.05).  Table 4 displays the comparison of liver function recovery. The results presented that probiotics helped to promote the recovery of liver function.

## 4. Discussion

Traditionally, bowel preparation was considered as a pivotal part of preoperative nursing work for partial hepatectomy, which was beneficial to reduce postoperative infection caused by intestinal flora translocation [19]. Although mechanical bowel preparation (MBP) is generally used for partial hepatectomy [20], it has been questioned in recent years. Hokuto et al. [20] compared the perioperative outcomes of patients who received or did not receive MBP before liver resection, and they manifested that the use of MBP has no significant effect on short-term outcomes after liver resection in patients with hepatocellular carcinoma (HCC); therefore, liver surgery can omit MBP. To sum up, MBP could not provide effective benefits to patients before liver surgery, and drinking plenty of water and diarrhea significantly increased the discomfort at preoperative preparation. Therefore, our patients were not treated with MBP according to current guidelines and research results.

The article "Influences of Oral Administration of Probiotics on Posthepatectomy Recovery in Patients in Child-Pugh Grade" was published in 2022. Journal: Comput Math Methods Med.

It is well known that HCC is generally the last stage of the development of chronic liver disease, and liver resection is the preferred treatment for most patients [21]. But surgical stress induces dysbiosis, promotes the release of inflammatory cytokines, and increases the permeability of the intestinal barrier, leading to bacterial translocation [21, 22]. The liver is exposed to microbiota and microbial metabolites through portal flow, which ultimately leads to increased infection and poor prognosis due to the limited detoxification function of the liver [21, 23]. The bidirectional relationship between the gut with its microbiota and the liver is known as the “gut-liver axis” [24]. The gut microbiota, as a key factor in this axis, contributes to the progression of liver disease at different stages, thereby promoting the development of HCC and can be used as a noninvasive biomarker for the disease [25–27]. Hence, maintaining intestinal homeostasis is pivotal.

Consideration attention has been given to physiopathological significance of gut microbiota and gut microecological balance, which lays a theoretical basis for rational bowel preparation methods [24]. Probiotics, which can prevent bacterial translocation by stabilizing the intestinal barrier and stimulating the proliferation, mucus secretion, and motility of the intestinal epithelium, have been suggested as a treatment for different types of chronic liver injury [28, 29]. In a randomized controlled trial, daily intake of a probiotic preparation (VSL#3) is found to significantly reduce the risk of hospitalization in patients with hepatic encephalopathy, as well as the Child-Turcotte-Pugh and end-stage liver disease (MELD) scoring model [30]. Alisi et al. [31] also demonstrated that taking a VSL#3 supplement notably improves NAFLD in children. A meta-analysis illustrated that a combination of probiotics and prebiotics given to patients before or on the day of liver transplantation noticeably reduces postoperative infection rates and antibiotic use compared with patients in the prebiotic-only group [29]. Additionally, using probiotics in animal HCC models can alleviate gut dysbiosis and produce anti-inflammatory mediators to repress tumor growth [32]. Clinically, Rifatbegovic et al. [33] emphasized that cirrhotic HCC patients who took probiotics before and after surgery had faster recovery of liver function and fewer complications. Meanwhile, taking probiotics aids in reducing morbidity and mortality. Furthermore, preoperative application of probiotics to modulate intestinal flora is deemed as a functional bowel preparation strategy, and it has achieved better postoperative recovery results than MBP in patients with colon cancer surgery, pancreaticoduodenectomy, and electroprostatectomy [34–36]. But no study has reported the impact of preoperative probiotic administration on infection and liver function recovery after partial hepatectomy in patients with different Child grades.

The article "Influences of Oral Administration of Probiotics on Posthepatectomy Recovery in Patients in Child-Pugh Grade" was published in 2022. Journal: Comput Math Methods Med.

Clostridium butyricum is a type of probiotics, whose pharmacological effects are as follows: Clostridium butyricum can facilitate the growth of beneficial bacteria in the intestine and repress the reproduction of harmful bacteria. Its metabolites can facilitate the repair and regeneration of intestinal epithelium and restore and maintain the intestinal microecological balance. In addition, its metabolites can also correct intestinal flora alternation and repress the overgrowth of G-bacteria and bacterial translocation, thereby reducing intestinal permeability and restoring intestinal mucosal barrier [37]. One study unveiled that Clostridium butyricum could reduce generation and release of endotoxin in acute hepatic failure and relieve IETM, thereby reducing the secondary lesion of liver tissue. Moreover, butyric acid produced by Clostridium butyricum can effectively constrain the transfer of nuclear factor kappa B (NF-*κ*B) into the nucleus while repressing the binding of NF-*κ*B and DNA, thus restraining gene expression of a series of proinflammatory factors such as TNF-*α* and exerting effective effects on the treatment of liver disease [38]. Clinical study indicated that intestinal barrier and liver function in patients with liver cirrhosis could be effectively improved by using Clostridium butyricum [39]. Hence, Clostridium butyricum has been proved to be an effective agent against infection and hepatic injury in patients with chronic liver disease. In this study, we manifested that probiotics markedly reduced calcitonin content in the Child-Pugh B grade subgroup on postoperative day 3 and day 5, indicating that probiotics could reduce early postoperative bacterial infections. In addition, probiotics also noticeably decreased the content of ALT in the Child-Pugh B grade subgroup, while reducing PT, indicating that probiotics can accelerate the recovery of liver function. But in the Child-Pugh A grade subgroup, probiotics had no notable effect on infection markers, liver function markers, or coagulation markers. Patients in the Child-Pugh A grade subgroup may not present obvious intestinal flora disturbance due to mild liver disease, while most of the patients in Child-Pugh B grade subgroup have a long history of liver disease with significant intestinal flora disturbance. Thus, prominent differences exist in patients' response to treatment with probiotic preparations.

The article "Influences of Oral Administration of Probiotics on Posthepatectomy Recovery in Patients in Child-Pugh Grade" was published in 2022. Journal: Comput Math Methods Med.

This study may be somewhat limited as a single-center study with the small sample size. Further verification by a multicenter study with large sample size is warranted. Additionally, we will perform liver cancer classification based on a multicenter large sample to observe whether probiotics in different types of liver cancer also work best in Child-Pugh B grade patients. Besides, mechanisms and detection of intestinal flora are still underexplored.

To sum up, the value of probiotics in the treatment of liver disease was verified previously. In this research, a subgroup analysis of infection and liver function after partial hepatectomy and oral probiotics in patients with different Child-Pugh grades was carried out. The results illustrated that patients in the Child-Pugh A grade subgroup did not benefit from oral probiotics. But patients in Child-Pugh B grade subgroup had fewer postoperative infections and accelerated recovery of liver function. This study provides a basis for the improvement and individualized application of bowel preparation measures in patients who underwent hepatectomy and unravels the clinical effect of oral probiotics in improving postoperative infection and liver function recovery in those patients.

## Figures and Tables

**Table 1:** Child-Pugh score.

Parameter	Score		
	1 point	2 points	3 points
Hepatic encephalopathy	None	1-2	3-4
Ascites	None	Mild	Moderate or severe
Serum total bilirubin (TBIL) (*μ*mol/L)	<34	34-51	>51
Serum albumin (ALB) (g/L)	≥35	28-35	<28
Prothrombin time (PT) (s)	≤14	15-17	≥17

Grade A = 5-6 points; grade B = 7-9 points; grade C = 10-15 points.

**Table 2:** Baseline information of patients.

	Child-Pugh A grade		*P* value	Child-Pugh B grade		*P* value
	Probiotics group (*n* = 25)	Control group (*n* = 25)		Probiotics group (*n* = 25)	Control group (*n* = 25)	
Sex						
Male	19	21	0.480	20	23	0.221
Female	6	4		5	2	
Age						
≥60 years	13	12	0.777	10	12	0.569
<60 years	12	13		15	13	
Body mass index (BMI)	23.34 ± 0.36	23.53 ± 0.85	0.309	24.32 ± 0.74	24.39 ± 0.96	0.774
Liver cirrhosis						
Yes	5	4	0.713	20	21	0.713
No	20	21		5	4	
Serum TBIL (*μ*mol/L)	17.23 ± 2.34	16.64 ± 0.56	0.226	23.23 ± 4.87	24.09 ± 3.56	0.479
Serum ALB (g/L)	38.34 ± 0.40	38.50 ± 0.55	0.245	33.10 ± 0.75	33.50 ± 0.83	0.080
PT (s)	11.36 ± 0.39	11.54 ± 0.32	0.081	12.20 ± 0.63	12.54 ± 0.92	0.134
Serum creatinine (*μ*mol/L)	66.21 ± 2.34	65.21 ± 4.21	0.053	70.21 ± 5.09	71.43 ± 3.02	0.244
Resecting more than 30% of the liver						
Yes	14	11	0.396	10	16	0.089
No	11	14		15	9	

The article "Influences of Oral Administration of Probiotics on Posthepatectomy Recovery in Patients in Child-Pugh Grade" was published in 2022. Journal: Comput Math Methods Med.

**Table 3:** Comparison of infection indexes of patients.

	Child-Pugh A grade		*P* value	Child-Pugh B grade		*P* value
	Probiotics group (*n* = 25)	Control group (*n* = 25)		Probiotics group (*n* = 25)	Control group (*n* = 25)	
Procalcitonin (ng/mL)						
Day 1 after surgery	1.94 ± 7.29	1.28 ± 2.08	0.665	4.33 ± 11.77	4.09 ± 11.78	0.943
Day 3 after surgery	1.49 ± 3.72	1.41 ± 2.91	0.933	0.80 ± 0.96	1.98 ± 1.88	0.007
Day 5 after surgery	0.75 ± 1.25	0.51 ± 0.86	0.433	0.29 ± 0.47	1.14 ± 1.59	0.014
Limulus test for endotoxins (Eu/mL)						
Day 1 after surgery	0.11 ± 0.19	0.13 ± 0.21	0.726	0.27 ± 0.45	0.16 ± 0.24	0.286
Day 3 after surgery	0.21 ± 0.43	0.15 ± 0.27	0.534	0.17 ± 0.39	0.22 ± 0.39	0.652
Day 5 after surgery	0.16 ± 0.16	0.15 ± 0.18	0.836	0.22 ± 0.53	0.41 ± 0.78	0.319
Interleukin-6 (pg/mL)						
Day 1 after surgery	153.20 ± 437.00	144.20 ± 165.80	0.924	135.40 ± 116.20	155.30 ± 103.20	0.525
Day 3 after surgery	106.80 ± 173.50	81.24 ± 88.14	0.515	97.52 ± 119.60	94.94 ± 105.30	0.936
Day 5 after surgery	48.25 ± 53.45	46.41 ± 45.38	0.896	34.65 ± 30.77	28.99 ± 16.43	0.421

**Table 4:** Comparison of liver function indexes of patients.

	Child-Pugh A grade		*P* value	Child-Pugh B grade		*P* value
	Probiotics group (*n* = 25)	Control group (*n* = 25)		Probiotics group (*n* = 25)	Control group (*n* = 25)	
Serum ALT (U/L)						
Day 1 after surgery	288.30 ± 196.20	271.30 ± 183.70	0.753	258.80 ± 253.50	254.90 ± 181.80	0.950
Day 3 after surgery	108.50 ± 77.33	113.70 ± 91.00	0.829	115.30 ± 79.56	216.20 ± 184.1	0.015
Day 5 after surgery	69.86 ± 37.49	75.58 ± 48.91	0.645	90.28 ± 61.36	138.80 ± 78.28	0.019
Serum TBIL (*μ*mol/L)						
Day 1 after surgery	23.99 ± 18.33	23.70 ± 13.75	0.950	25.34 ± 29.23	24.80 ± 9.65	0.931
Day 3 after surgery	21.23 ± 19.79	21.78 ± 9.19	0.900	23.75 ± 15.97	23.57 ± 8.89	0.961
Day 5 after surgery	18.92 ± 15.79	19.84 ± 8.36	0.798	20.00 ± 12.50	23.37 ± 11.21	0.321
PT (s)						
Day 1 after surgery	12.82 ± 1.609	13.06 ± 1.416	0.579	12.63 ± 1.28	12.92 ± 1.08	0.391
Day 3 after surgery	12.33 ± 1.369	12.96 ± 1.311	0.103	12.50 ± 1.40	13.63 ± 1.56	0.010
Day 5 after surgery	11.99 ± 2.292	12.82 ± 1.358	0.126	11.38 ± 2.736	12.79 ± 1.116	0.021

## Data Availability

The date and materials in the current study are available from the corresponding author on reasonable request.
